The article "Film Effect Optimization by Deep Learning and Virtual Reality Technology in New Media Environment" was published in 2022. Journal: Comput Intell Neurosci.

# Film Effect Optimization by Deep Learning and Virtual Reality Technology in New Media Environment

**DOI:** 10.1155/2022/8918073

**Published:** 2022-05-20

**Authors:** Linlin Cui, Zhuoran Zhang, Jiayi Wang, Zhu Meng

**Affiliations:** ^1^Department of Directing, Qingdao Film Academy, Qingdao City 266000, China; ^2^Department of Media, Arts and Humanities, University of Sussex, Brighton BN1 9RH, UK

## Abstract

Today, new media technology has widely penetrated art forms such as film and television, which has changed the way of visual expression in the new media environment. To better solve the problems of weak immersion, poor interaction, and low degree of simulation, the present work uses deep learning technology and virtual reality (VR) technology to optimize the film playing effect. Firstly, the optimized extremum median filter algorithm is used to optimize the “burr” phenomenon and a low compression ratio of the single video image. Secondly, the Generative Adversarial Network (GAN) in deep learning technology is used to enhance the data of the single video image. Finally, the decision tree algorithm and hierarchical clustering algorithm are used for the color enhancement of VR images. The experimental results show that the contrast of a single-frame image optimized by this system is 4.21, the entropy is 8.66, and the noise ratio is 145.1, which shows that this method can effectively adjust the contrast parameters to prevent the loss of details and reduce the dazzling intensity. The quality and diversity of the specific types of images generated by the proposed GAN are improved compared with the current mainstream GAN method with supervision, which is in line with the subjective evaluation results of human beings. The Frechet Inception Distance value is also significantly improved compared with Self-Attention Generative Adversarial Network. It shows that the sample generated by the proposed method has precise details and rich texture features. The proposed scheme provides a reference for optimizing the interactivity, immersion, and simulation of VR film.

## 1. Introduction

Since 2000, the development of new media has shown good momentum. By 2013, new media entered a particular stage of development: the apparent globalization, communication, networking, mobility, and social integration of new media. Social and group communication are increasingly open and connected through new media [1,2]. Based on this situation, new media's cultural and entertainment functions continue to expand. With the terminal revolution of smartphones and tablet computers, new media has increasingly become a cultural and entertainment platform. The visual marketing and coping strategies of art forms and film titles and changes in audience acceptance are necessary under the new wave of multimedia technology. Using technology to improve the film market is the core of our discussion [3].

The article "Film Effect Optimization by Deep Learning and Virtual Reality Technology in New Media Environment" was published in 2022. Journal: Comput Intell Neurosci.

Researchers have carried out a lot of research in related fields. Zhang and Min (2020) [4] optimized and simulated the visual effect of garden graphics by using the Particle Swarm Optimization (PSO) algorithm and Wavelet Threshold algorithm. To make up for the deficiency of the activation function of the Deep Belief Network (DBN), the author used the wavelet function as the activation function of DBN to improve the recognition accuracy. The experimental results showed that the hybrid optimization algorithm of the Genetic Algorithm and PSO algorithm had the best classification effect. Jalab et al. (2021) [5] noted that medical image enhancement was a challenging research task. Therefore, the authors proposed a new fractional integral entropy for estimating the unpredictable probability of image pixels. Overall, their optimized model improved the details of Magnetic Resonance Imaging (MRI) scan of brains, Computerized Tomography scan of lungs, and MRI scan of kidneys. Feng et al. (2020) [6] reported that existing image enhancement techniques were prone to loss of details, resulting in local under- or overexposure, as well as color distortion, and failed to balance contrast and color fidelity. The authors proposed a color image enhancement algorithm based on adaptive weighted Retinex and wavelet transform to solve these problems. This algorithm converted the image from red, green, and blue (RGB) space to hue saturation intensity space. It decomposed the luminance component intensity into low-frequency luminance images and multiple high-frequency luminance images by wavelet. They also performed adaptive weighted Retinex enhancement on low-frequency photos and improved the threshold for high-frequency image denoising. Finally, the inverse wavelet transform was used to reconstruct the luminance component. After gamma correction, the contrast was further enhanced and converted to RGB space for an improved image. The experimental results indicated that the algorithm effectively enhanced the contrast and color fidelity of the image and preserved the details and texture of the picture. Sen and Rout (2020) [7] studied the detection and removal of noisy pixels in impulse noise-contaminated images. They proposed a noise detection method to avoid noiseless pixels being mistaken for noise and an improved pruned median filter algorithm based on probabilistic decisions to resolve conflicts associated with an even number of noise-free pixels in pruned median filters. Simulation results proved that the algorithm could detect and contaminate images and had good visual expressiveness. Wang et al. (2021) [8] believed that the primary purpose of image enhancement technology was to improve image quality; however, existing enhancement algorithms were prone to overexposure and incorrect detail processing. The authors proposed an image enhancement algorithm based on fractional order and relative total variation. The algorithm removed the noise in the original image by low-pass filtering, extracted the edge of the image with fractional order, and then fused the image with the extracted edge through the fractional order. Finally, the authors conducted several experiments to verify the effect of the algorithm on different data sets. Li et al. (2021) [9] put forward a traffic image enhancement model based on illumination adjustment and depth difference. The algorithm used the dark channel principle to obtain the image's depth of field and employed the spectral clustering algorithm to cluster the image's depth of field. The experimental results suggested that the model could effectively enhance the uneven illumination and haze weather images in traffic scenes, achieve excellent visual effects, generate rich details, and improve the quality of traffic images, meeting the needs of practical traffic applications. In the branch of image enhancement technology in the research of movie picture optimization, the remaining research difficulties can be divided into the following two points. First, the quality of the generated image is poor, the detailed information is imperfect, and the definition is not high. Second, the model's training is challenging, and it has massive parameters and insufficient generalization ability.

The article "Film Effect Optimization by Deep Learning and Virtual Reality Technology in New Media Environment" was published in 2022. Journal: Comput Intell Neurosci.

Here is the significance of the present research. In today's society, “high virtual ecology” created by “virtual reality (VR) + content” has covered many fields such as video games, live activities, video entertainment, medical treatment, real estate, retail, education, engineering, and military. The “marriage” between film and VR in video entertainment has the most inherent advantages. For a long time, the shocking audiovisual effect pursued by the film industry has a solid inertial dependence on cutting-edge technology. The effect experience of VR is highly consistent with the immersion and exclusivity of film art itself. Therefore, VR film has received extensive attention from the beginning of its birth. As a highly innovative media form, VR film has constructed a revolutionary visual image presentation mode and a new aesthetic space with immersion, interaction, and simulation characteristics. At the same time, the booming film industry has also accelerated the upgrading of VR technology. The development of film art is closely related to the technical level, opening up a new era in film and creating a new form of film. In the digital age, the connection between film and TV technology is closer, especially in the application of magic films and science fiction films. VR technology can create a new audiovisual effect, which is more infectious and artistic innovation than general film art. The combination of art and technology is the trend of modern and contemporary social and cultural development. Technology and art complement each other and develop together. VR creates a new film-viewing experience through interactive, immersive, and imaginative features, effectively improving the film's visual impact. Last but not least, VR technology is of great significance in combining real data information and virtual environment data information. It promotes the transformation and upgrading of film technology and revolutions of the traditional film-viewing mode. It provides a completely different film-viewing experience for the audience.

The article "Film Effect Optimization by Deep Learning and Virtual Reality Technology in New Media Environment" was published in 2022. Journal: Comput Intell Neurosci.

The following is the innovation and contribution of the present work. Firstly, the threshold is added to construct the extremum median filter algorithm to enhance the image pixel sorting of the filter window. Through prejudgment, the image area is divided into image edge, flat, and noisy areas. The second point is to optimize the Generative Adversarial Network (GAN) and use the optimized image to enhance the data of the single video image. Lastly, it uses a decision tree and hierarchical clustering algorithm for VR image color enhancement. The proposed algorithm completes the image enhancement task better than the other literature methods.

The research is organized as follows. The “Introduction” briefly explains the new media technology and movie image optimization technology. VR technology in movies is explored in “Research on the application of VR technology in movies.” The image preprocessing technology is researched and optimized. An improved GAN image enhancement algorithm is proposed alongside the image color enhancement technology based on the optimized decision tree. The experimental results are explained in “Analysis of experimental results.” Lastly, the experimental results are encapsulated in “Conclusions.”

## 2. Research on the Application of VR Technology in Movies

### 2.1. Application Analysis of Virtual Reality Technology in Film

In 1977, digital virtual imaging technology was applied to the film Star Wars by American director George Lucas. In March 1993, the VR technology represented by Jurassic Park entered a stage of rapid development, marking the beginning of a new digital virtual era for films globally [10–12]. VR film immersion is derived from the audience's subjective projection of film characters, the deep resonance with the film plot, and the subconscious identification of emotional ethics. It is also the product of the viewers' knowledge-seeking initiative at the human-computer interaction (HCI) level.

The article "Film Effect Optimization by Deep Learning and Virtual Reality Technology in New Media Environment" was published in 2022. Journal: Comput Intell Neurosci.

VR technology can also simulate the “characters” and “scenes” in life and reproduce real actors' facial expressions and performance actions. There are strict requirements for photographic equipment in traditional film shooting, and the shooting range is only focused on the lens. By comparison, VR technology can provide a corner-covering and full-scene shooting approach. Meanwhile, deviation during shooting can also be adjusted easily through postproduction. At present, performance capture technology has been promoted in film production. Performance capture combines computer animation and real-life performance to generate close-to-real-life expression and shape. The core equipment is face capture headgear. Actors need to wear miniature high-definition camera equipment when performing. The equipment can capture actors' facial movements with high accuracy of 95%, thus making them extremely clear compared with traditional photography [13, 14]. The representative film is Final Fantasy: The Spirit Within (2001). VR technology can visualize a role, real or imagined, in front of the audience and improve the film's attraction [15, 16].

Contemporary new visual culture is born with the development of science and technology, which has a fatal impact on the traditional film culture. In recent years, the proportion of films actors-centered has decreased year by year, and the proportion of three-dimensional (3D) images is catching up swiftly. The 3D images created by virtual TV technology can better set off the film's emotion and improve the film's artistic expression. In terms of types, 3D films feature three categories. (1) Suspense: the suspense scene created by VR technology is unmatched by traditional technology. Suspense scenes promote the plot development and feed the audiences' curiosity. (2) Sense of crisis: VR technology can also create exaggerated images and simulate intuitive images imagined to convey the emotion of a sense of crisis. For example, in the film 2012 (2009), more than 1,000 special effects lenses are used to create virtual scenes, showing the scenes of sea floods, mountain collapses, and Earth cracks, which are very shocking. (3) Mystery: VR technology can also create mysterious images such as the fantasy planet picture in Avatar (2009). When such scenes are presented to the audience, they will naturally be attracted by this mysterious magical picture.

The article "Film Effect Optimization by Deep Learning and Virtual Reality Technology in New Media Environment" was published in 2022. Journal: Comput Intell Neurosci.

Figure 1 shows the application of VR in filmmaking.

Based on this, this paper uses VR image acquisition equipment to collect and summarize the real-time facial expression images of the audience. It relies on the accurate algorithms of machine learning technology to effectively identify the image data of facial expressions. Then, the VR control system can be targeted for fine-tuning to balance people's discomfort or enhance comfort. For example, the Convolutional Neural Network model can collect and classify the audiences' facial information when they have an emotional reaction due to the intensity of the movie sound or when the audiences' eyes deviate from the main plot. Then, the control system can adjust the VR device in time to enhance the light, shadow, or sound effect in the line of sight direction of the main plot and meet the audience's personalized immersion experience.

## 3. Research and Optimization of Image Preprocessing Technology

As we all know, an image is a kind of two-dimensional data that can only be stored in one dimension in memory. The quantization method is often used for video image digitization [17, 18]. This paper arranges the image data in *M*×*N* data groups and obtains an approximately continuous image *f*(*x*, *y*) by equidistant sampling. Then, the mathematical relationship shown in the following equation holds.

(1) $$\begin{array}{c} f\left(x,y\right)=\left[\begin{array}{cccc} f\left(0,0\right) & f\left(0,1\right) & \cdots & f\left(0,M-1\right)\\ f\left(1,0\right) & f\left(1,1\right) & \cdots & f\left(1,M-1\right)\\ \cdots & \cdots & \cdots & \cdots \\ f\left(N-1,0\right) & f\left(N-1,1\right) & \cdots & f\left(N-1,M-1\right) \end{array}\right]. \end{array}$$

Each element in (1) represents a discrete variable.

Suppose that *x* and *y* in (1) represent real integers in the set z and *f*(*x*) is a function of assigning gray values to the point *f*(*x*, *y*). Then, *f*(y) represents a complete spatial digitized image, and the assignment process is called the quantization process [8,9,19]. The image digitization process determines the size *M* and *N* of the processed image and the discrete grayscale count *G* of the pixel. (2) indicates the image digitization processing.

(2) $$\begin{array}{c} \left\{\begin{array}{c} M=2^{m},\\ N=2^{n},\\ G=2^{k}. \end{array}\right. \end{array}$$

The principle of median filtering is to replace the value of a point in the digital image with the median value in the neighborhood of the point. The median value is calculated as follows.

This paper defines a set of data as *x*_1_, *x*_2_, *x*_3_,…, *x*_*n*_ and arranges these *n* values in numerical order. Then, there is the mathematical relationship shown in the following equation:

(3) $$\begin{array}{c} x_{il}⩽x_{i2}⩽x_{i3}⩽\cdots ⩽x_{\text{in}}. \end{array}$$

When *n* in (3) is an odd number, there is a mathematical relationship presented in the following equation:

(4) $$\begin{array}{c} y=Med\left(x_{1},x_{2},x_{3},\ldots ,x_{n}\right)\\ =x_{i}\frac{\left(n+1\right)}{2}. \end{array}$$

When *n* in (3) is an even number, there is a mathematical relationship shown in the following equation:

(5) $$\begin{array}{c} y=Med\left(x_{1},x_{2},x_{3},\ldots ,x_{n}\right)\\ =\frac{1}{2}\left[x_{i}\frac{\left(n+1\right)}{2}+x_{i}\frac{\left(n\right)}{2}+1\right]. \end{array}$$

According to the calculation results of the above equations, the image median filtering effect is similar to the result obtained by the simple neighborhood average method under the 3 × 3 window. Here, *x*(*m*, *n*) is described as the original video image mixed with noise and the gray value of the pixel at the coordinates of (*m*, *n*). First, a rectangular window is selected and denoted as *L*=2*N*+1, where N represents a nonnegative integer. This window is divided into four equal subwindows. The process is described as

(6) $$\begin{array}{c} W_{1}\left(m,n\right)=\left\{x\left(m,n+i\right),\;-N⩽i⩽N\right\},\\ W_{2}\left(m,n\right)=\left\{x\left(m+i,n\right),\;-N⩽i⩽N\right\},\\ W_{3}\left(m,n\right)=\left\{x\left(m+i,n-i\right),\;-N⩽i⩽N\right\},\\ W_{4}\left(m,n\right)=\left\{x\left(m+i,n-i\right),\;-N⩽i⩽N\right\}. \end{array}$$

*W*_1_, *W*_2_, *W*_3_, and *W*_4_ represent one-dimensional image windows rotated horizontally or vertically. Let *Z*_1_(*m*, *n*), *Z*_2_(*m*, *n*), *Z*_3_(*m*, *n*), and *Z*_4_(*m*, *n*) be the median values of the four windows, which can be described as

(7) $$\begin{array}{c} Z_{1}\left(m,n\right)=med\left[x\left(i,J\right)\in W_{1}\left(m,n\right)\right],\\ Z_{2}\left(m,n\right)=med\left[x\left(i,j\right)\in W_{2}\left(m,n\right)\right],\\ Z_{3}\left(m,n\right)=med\left[x\left(i,j\right)\in W_{3}\left(m,n\right)\right],\\ Z_{4}\left(m,n\right)=med\left[x\left(i,j\right)\in W_{4}\left(m,n\right)\right]. \end{array}$$

Denote *U*_max_(*m*, *n*) and *U*_max_(*m*, *n*) as the maximum value and the minimum value among the *Z*_1_(*m*, *n*), *Z*_2_(*m*, *n*), *Z*_3_(*m*, *n*), and *Z*_4_(*m*, *n*). Then, there is a mathematical relationship shown in the following equations:

(8) $$\begin{array}{c} U_{\max}\left(m,n\right)=\max\left[Z_{1}\left(m,n\right),Z_{2}\left(m,n\right),Z_{3}\left(m,n\right),Z_{4}\left(m,n\right)\right], \end{array}$$

(9) $$\begin{array}{c} U_{\min}\left(m,n\right)=\min\left[Z_{1}\left(m,n\right),Z_{2}\left(m,n\right),Z_{3}\left(m,n\right),Z_{4}\left(m,n\right)\right]. \end{array}$$

According to (8) and (9), the output form of the single-term multistage median filter can be written as

(10) $$\begin{array}{c} y\left(m,n\right)=med\left[U_{\min}\left(m,n\right),U_{\max}\left(m,n\right),x\left(m,n\right)\right]. \end{array}$$

Here, an extreme median filtering algorithm is constructed by adding thresholds to enhance the image pixel sorting ability of the filtering window. The image area is divided into image edge detail area, flat area, and noise affected area by prejudgment. The optimization process is as follows.

The article "Film Effect Optimization by Deep Learning and Virtual Reality Technology in New Media Environment" was published in 2022. Journal: Comput Intell Neurosci.

First, the pixels in the window max(*W*[*x*_*i*,*j*_]) are sorted to find the points [*x*_*i*,*j*_] and min(*W*[*x*_*i*,*j*_]), that is, the maximum and minimum points. Then, the point *x*_*ij*_ is compared with the max(*W*[*x*_*i*,*j*_]) and min(*W*[*x*_*i*,*j*_]). According to the comparison result, if *x*_*ij*_ is an extremum point, the original value will be transmitted without filtering; otherwise, the prejudgment algorithm will be used for processing. *f*(*x*, *y*) is set as the gray value of the image point (*x*, *y*), and g(*x*, *y*) is set as the gray value of the neighborhood point of (*x*, *y*). An operator *Y* is chosen to act on g(*x*, *y*) and *f*(*x*, *y*), and it comes to *Y*=*Y*(*f*, *g*). Then, the subsequent operations are based on different values of *Y*, which can be expressed as

(11) $$\begin{array}{c} Y=\sum_{i=0}^{T}y\left(f\left(x,y\right)-g_{i}\left(x,y\right)\right). \end{array}$$

(11) can be transformed into

(12) $$\begin{array}{c} Y\left(x\right)=\left\{\begin{array}{cc} 1 & \left|x\right|⩽T,\\ 0 & \left|x\right|>T, \end{array}\right. \end{array}$$

where *T* stands for the time threshold.

## 4. Research on the Image Enhancement Algorithm Based on GAN

GAN is a new generative model network framework proposed by researcher Ian Goodfellow in 2014 based on the zero-sum game idea in game theory. The structure of GAN is mainly composed of two parts: the generator (*G*) network and the discriminator (*D*) network. The task of the *D* network is to distinguish the samples generated by *G* from the training data. The *G* network is responsible for confusing *D* by generating illustrations with a distribution close to the training data distribution [20–22]. The two learn the distribution of data by opposing each other, forming a dynamic “two-player min-max game”.  Figure 2 is the structural schematic diagram of the GAN model.

The image samples generated by GAN are of high quality and have good definitions. However, GAN currently has many disadvantages such as poor model interpretability. Besides, the distribution of the generated model is not explicitly expressed, which is challenging to train and prone to problems, such as gradient disappearance and mode collapse. Researchers add some conditional constraints to GAN and propose the Conditional Generative Adversarial Network (CGAN) [23,24]. In the *G* network of CGAN, the prior input noise and conditional information are combined to form a multimodal vector, which is sent to the *G* network as input representation information. The category label is introduced into the discriminant network as a conditional variable. If false, it is also necessary to judge whether the generated category matches the category of the input image.  Figure 3 represents the network structure of CGAN [25,26].

The article "Film Effect Optimization by Deep Learning and Virtual Reality Technology in New Media Environment" was published in 2022. Journal: Comput Intell Neurosci.

The objective function of CGAN is a two-player max-min game with conditional probability. The prior probability distribution *D*(*x*),*G*(*z*) of CGAN is transformed into the corresponding posterior probability distribution *D*(*x|c*),*G*(*z|c*) as shown in the following equation:

(13) $$\begin{array}{c} \min_{G}\max_{D}V\left(D,G\right)=E_{x-p_{\text{dutu}}\left(x\right)}\left[\log\;D\left(x|c\right)\right]+E_{z-p_{z}\left(z\right)}\left[\log\left(1-D\left(G\left(z|c\right)\right)\right)\right]. \end{array}$$

The training method of CGAN is the same as that of GAN. Through alternating iterations of adversarial training, the optimizer performs the maximum and minimum operations to maximize the loss value of the discriminator [27] and minimize the loss value of the generator until they both stabilize.

The attention mechanism proposed by the visual image field has been widely used in various areas of deep learning. For instance, the applications of the attention mechanism include Spatial Attention and Temporal Attention. From the perspective of the role, the attention mechanism is divided into Soft Attention and Hard Attention. Hu et al. (2021) used the fuzzy system to study image prediction [28]. This paper employs the attention mechanism model in image generation applications to complete the task of data augmentation. The self-attention mechanism simply computes the response of a single location in the weighted sum of the features at all locations. This mechanism allows the network to focus on regions scattered but structurally related [29–31].  Figure 4 illustrates the self-attention module in Soft Attention Generative Adversarial Network (SAGAN).

The network model shown in Figure 4 is the feature map *x* of the convolution calculated by the hidden layer of the convolutional network. Then, the two feature spaces *f*=*W*_*f*_*x* and *g*=*W*_*g*_*x* are obtained through the convolution kernel 1 × 1. *f* and *g* are used to calculate the attention. The specific calculation is given in (2).

(14) $$\begin{array}{c} \beta_{j,i}=\frac{\exp\left(s_{ij}\right)}{\sum_{i=1}^{N}\exp\left(s_{ij}\right)},\\ s_{ij}=f{\left(x_{i}\right)}^{T}g\left(x_{j}\right). \end{array}$$

This paper uses the supervision idea of CGAN to introduce conditional variables into the generator and discriminator to solve the problem of specifying categories of generated images. Additional guidance information is used to generate corresponding data. Then, the self-attention mechanism is introduced into the SAGAN model.  Figure 5 shows the framework of the model reported here.

The article "Film Effect Optimization by Deep Learning and Virtual Reality Technology in New Media Environment" was published in 2022. Journal: Comput Intell Neurosci.

## 5. Research on the Image Color Enhancement Technology Based on the Optimal Decision Tree Algorithm

In VR movies, controlling professional equipment through body movements is more maneuverable, faster, and better than facial expressions. This paper first collects human gestures and posture images to efficiently complete the process of human action feature extraction, motion capture, action tracking, etc. Then, some machine learning technologies are cross-combined for mutually complementing superiority to efficiently identify and process the real-time image data of these body movements, including the Back Propagation (BP) Neural Network, Features from Accelerated Segment Test (FAST), Speeded Up Robust Feature (SURF) algorithm, Support Vector Machine (SVM), and K-Nearest-Neighbor (KNN). In this way, VR controlling equipment can receive and respond to signals more accurately and timely to provide audiences with a personalized interactive experience with deep interaction and robust control [32,33]. First, the FAST algorithm and the stable SURF algorithm are used to extract the features of the posture and gesture images, respectively. Secondly, the posture and gesture features are classified by the SVM and KNN algorithms, respectively. The BP neural network is used to optimize the threshold space in the FAST algorithm and the K value space in the KNN algorithm. Optimizing the threshold and K value can also ensure the efficient operation of the recognition rate. Then, the human body posture and gesture features are recognized and matched. Finally, the interaction results are transmitted to the VR system.  Figure 6 shows the structure of the BP Neural Network.  Figure 7 reveals the optimization model under the decision tree and hierarchical clustering algorithm.

The model construction process is divided into three steps. (1) Cluster analysis clusters the image frames with the same quality in a film using the system clustering method to form several intervals as the classification target of the decision tree model. (2) Influencing factor index system is established by finding factors affecting image quality, including external and internal factors. (3) The decision tree model is implemented by inputting the attribute vector corresponding to the influencing factors into the decision tree model. The decision tree is classified and trained based on the clustering interval of picture frame quality. Through the above algorithm, the image of the character can be changed.

The article "Film Effect Optimization by Deep Learning and Virtual Reality Technology in New Media Environment" was published in 2022. Journal: Comput Intell Neurosci.

## 6. Configuration of Software and Hardware Environment and Model Parameters

This experiment uses a personal server. The CPU is Intel (*R*) Xeon (*R*) CPU e5-2620 V4 @ 2.10 GHz. The hard disk is 2T SSD. The GPU is NVIDIA Tesla P100, the video memory configuration is 16 GB, and the operating system configuration is windows10. Besides, CUDA 9.0, Python 3.6, and TensorFlow 1.9.0 are adopted. The development tool is PyChart.

The adaptive learning rate algorithm Adam is selected as the optimizer in the training model, where the parameter beta 1 is set to 0.5, and beta 2 is set to 0.9. The required hyperparameters in the model include batch_size (the number of samples per batch), set to 64.

## 7. Analysis of Experimental Results

### 7.1. Analysis of Optimization Results of the Median Filter Algorithm

The VR-based video image optimization simulation system proposed here is compared with the image processing methods based on the simulation system, digital signal processing (DSP), and field-programmable gate array (FPGA).  Figure 8 provides the simulation results.

According to Figure 8, the processing effect of this algorithm is the best because the algorithm in this paper can calculate the most applicable threshold value. Although other algorithms can achieve the optimization purpose, they cannot achieve satisfactory results. The reason may be that the image optimization standard value is difficult to calculate.

Figure 9 shows the comparison results of the algorithm performance.

The contrast of picture (a) in Figure 8 is 2.45, the entropy is 9.33, and the noise ratio is 48.7. The contrast of the image (c) in Figure 8 is 12.45, the entropy is 11.33, and the noise ratio is 189.2. The contrast of picture (f) in Figure 8 is 4.21, the entropy is 8.66, and the noise ratio is 145.1. The contrast, entropy, and noise of the images processed by the algorithm reported here are lower than other methods. These results prove that this method can effectively adjust the contrast parameters, prevent the loss of details, and reduce the intensity of glare.

The VR-based video image processing effect optimization simulation system proposed here is compared with the simulation system, DSP-based, and FPGA-based video image processing methods in high-brightness images. The simulation results are shown in Figure 10.

The article "Film Effect Optimization by Deep Learning and Virtual Reality Technology in New Media Environment" was published in 2022. Journal: Comput Intell Neurosci.

Figure 11 shows the comparison of the experimental results of different algorithms on images with higher brightness.

The contrast of picture (a) in Figure 10 is 2.25, the entropy is 8.33, and the noise ratio is 46.7. The contrast of picture (b) in Figure 11 is 10.45, the entropy is 19.33, and the noise ratio is 164.2. The contrast, entropy, and noise of the algorithm in this paper are all lower than other methods, indicating that this method can effectively adjust the contrast parameters, prevent the loss of details, and reduce the intensity of glare.

### 7.2. Comparison of the Experimental Results of the Optimized GAN

Figure 12 displays the samples generated by adding conditional features using the GAN model constructed here on the MNIST database.

It can be seen from Figure 12 that the model can learn accurate features after five iterations, but the image is noisy, and the details of the image are defective. After 30 iterations, the details of the sample image generated by the model are precise, diverse, and distinctive.

Figure 13(a) shows the changing trend of the discriminator loss function, and Figure 13(b) presents the changing trend of the generator loss.

According to Figure 13(a), the loss value decreases rapidly and vertically at the beginning of 1,000 iterations. After 2000 iterations, the loss value is relatively stable. In the subsequent iterations, the discriminator and the generator learn from each other so that the generated sample quality resolution is higher and the smoothness is better. Figure 13(b) indicates that after 1,500 iterations, the loss value of the generator increases gradually and steadily and tends to be stable. At this time, the loss of generator and discriminator tends to balance.

Figure 14 compares the model training under different learning rates.

It can be seen from Figure 14 that the loss value decreases fast when the initial learning rate is low and decreases more slowly when the learning rate is high. This shows that the initial learning rate is low, making the loss value drop rapidly. However, as the number of model iterations increases, the final loss value of the three learning rates decreases to the same level. However, the initial learning rate setting is relatively moderate, ensuring a faster training speed while ensuring better convergence.

The Frechet Inception Distance (FID) of the method proposed here is compared with that of other generative models, as shown in Table 1.

In Table 1, the FID values of the CGAN, Deep Convolution Generative Adversarial Network (DCGAN), Wasserstein Generative Adversarial Net (WGAN), SAGAN algorithm, and the algorithm reported here on the MNIST data set are 21.82, 18.82, 16.47, 10.41, and 9.21, respectively. The quality and diversity of specific types of images generated by the method proposed here are slightly improved compared to the current mainstream supervised GAN methods, which are in line with the subjective evaluation results of humans. Compared with SAGAN, the FID value is improved by 1.2.

The article "Film Effect Optimization by Deep Learning and Virtual Reality Technology in New Media Environment" was published in 2022. Journal: Comput Intell Neurosci.

Table 2 shows the comparison of optimization rates of various methods on the MNIST data set.

Under the same experimental conditions, the proposed method does not carry out image deskewing and normalization. However, the optimization rate is higher than the traditional methods. In the proposed model, the data enhancement effect by extracting features through confrontation training is better than preprocessing the original data.

## 8. Conclusions

Combining VR technology and film art has brought shocking visual effects to the audience, with more imaginative and artistic than traditional films. Therefore, this paper uses deep learning and VR technology to optimize the film playing effect. The research work can be divided into the following two points. First, it adds a threshold to the median filtering algorithm, constructs an extremum median filtering algorithm, enhances the image pixel sorting of the filtering window, and divides the image area into image edge, flat, and noisy areas through prejudgment. Then, it proposes a conditional self-attention GAN-based data enhancement method using supervised learning. Inspired by the idea of conditional GAN supervision, the network model introduces conditional variables into the generator and discriminator and uses additional information to guide the data generation process. The experimental results show that the proposed algorithm's contrast, entropy, and noise ratio are lower than other literature methods. Thus, the proposed method can effectively adjust the image contrast, prevent detail loss, and reduce the “burr” intensity. On the MNIST data set, the quality and diversity of the proposed method *r* to generate specific image types are slightly improved compared with the mainstream supervised GAN. The result is in line with the subjective evaluation results of human beings, and the FID is 1.2 higher than SAGAN.

Still, there are some deficiencies *i*. The network models used in this experiment are trained on a relatively simple neural network. The follow-up study will conduct in-depth research on the problems against the slow convergence speed of the generator and the discriminator in GAN. Meanwhile, a baseline measurement mechanism will be devised for the discriminator and generator for optimal model generation.

The article "Film Effect Optimization by Deep Learning and Virtual Reality Technology in New Media Environment" was published in 2022. Journal: Comput Intell Neurosci.

## Figures and Tables

**Figure 1:** Applications of VR technology in films: (a) a still from Star Wars; (b) a still from Jurassic Park; (c) application scenario of VR in Avatar.

**Figure 2:** Structure of the GAN model.

**Figure 3:** Structure of CGAN.

**Figure 4:** Structure of the attention mechanism module.

**Figure 5:** Schematic diagram of the model constructed here.

**Figure 6:** Structure of the BP neural network.

**Figure 7:** Optimization model under the decision tree and hierarchical clustering algorithm.

**Figure 8:** Comparison of the image optimization effects of different methods: (a) original image; (b) image after adding salt and pepper noise; (c) simulation system; (d) FPGA; (e) DSP; (f) the algorithm proposed here.

**Figure 9:** Algorithm performance comparison results: (a) the first test result; (b) the second test result.

**Figure 10:** Comparison of optimized processing for brighter images: (a) original image; (b) simulation system; (c) FPGA; (d) algorithm proposed in this paper.

**Figure 11:** Algorithm performance comparison results: (a) the first test result; (b) the second test result.

**Figure 12:** Samples generated vis the MNIST database: (a) epoch = 5; (b) epoch = 15; (c) epoch = 30; (d) epoch = 35.

**Figure 13:** Discriminator and generator loss trends: (a) discriminator; (b) generator.

**Figure 14:** Loss curves under three learning rates.

**Table 1:** Comparison of FID of different models.

Data set	CGAN	DCGAN	WGAN	SAGAN	The proposedmethod
CelebA	21.82	18.82	16.47	10.41	9.21

**Table 2:** Comparison of optimization rate.

Method	Pretraining	Optimization rate (%)
Linear classiﬁer	Deskewing	91.6
K-nearest-neighbors, euclidean	—	95
40 PCA (principal component analysis) + quadratic classiﬁer	—	96.2
SVM (support vector machin), Gaussian kernel	—	97.1
The proposed method	—	90

## Data Availability

The data used to support the findings of this study are included within the article.
